The article "Comparison of Diagnostic Value for Chronic Kidney Disease between 640-Slice Computed Tomography Kidney Scan and Conventional Computed Tomography Scan" was published in 2022. Journal: Contrast Media Mol Imaging.

# Comparison of Diagnostic Value for Chronic Kidney Disease between 640-Slice Computed Tomography Kidney Scan and Conventional Computed Tomography Scan

**DOI:** 10.1155/2022/6587617

**Published:** 2022-08-24

**Authors:** Yusen Zhao, Yaoyi Wang, Yuanbo Xu, Yijie Zhao, Yingwu Qu, Hua Zhang, Zhimin Zhang, Zhenshun Hu, Xiaolong Zhu, Shujun Cui, Jin Xie

**Affiliations:** ^1^Department of Medical Imaging, The First Affiliated Hospital of Hebei North University, Zhangjiakou City 075000, Hebei Province, China; ^2^Return Visit Center, The First Affiliated Hospital of Hebei North University, Zhangjiakou City 075000, Hebei Province, China; ^3^Library Information Department, Hebei North University, Zhangjiakou City 075000, Hebei Province, China; ^4^Medical Imaging Center, Central Hospital Affiliated to Shandong First Medical University, Jinan City 250013, Shandong Province, China

## Abstract

**Objective:**

To explore the diagnostic value for chronic kidney disease (CKD) between 640-slice computed tomography (CT) kidney scan and conventional CT scan.

**Methods:**

A total of 120 CKD patients who received kidney plain scan plus enhanced examination in the CT room of the Medical Imaging Department of our hospital from June 2019 to September 2019 were selected and randomly divided into the experimental group (*n* = 60) and the control group (*n* = 60). Patients in the control group received the conventional CT plain scan and enhanced scan, and for patients in the experimental group, CT plain scan was performed first, the range of 640-slice CT dynamic volume scan was determined, and after bolus injection of contrast agent, dynamic volume scan was performed for scanning in the cortical phase, myeloid phase, and secretory phase. The imaging quality and effective scanning dose were compared between the two modalities, and the relationship between CT values obtained from 640-slice CT scan and conventional CT scan and the renal impairment was analyzed.

**Results:**

Compared with the control group, the image quality of 640-slice CT scan conducted in the experimental group was significantly better (*P* < 0.05); the effective radiation doses of the experimental group and the control group were, respectively, (1.89 ± 0.32) mSv and (3.26 ± 0.47) mSv, indicating that the dose was significantly lower in the experimental group than in the control group (*t* = 18.664, *P* < 0.001), and the correlation analysis showed that the relationship between the sum of CT values in the cortical phase of both kidneys and kidney injury in the experimental group was *r* = 0.835, *P* < 0.001.

**Conclusion:**

Both 640-slice CT kidney scan and conventional CT scan can be used in the diagnosis of CKD. 640-slice CT has a lower radiation dose, better image quality, and higher application value.

## 1. Introduction

Chronic kidney disease (CKD) is a collective term for kidney diseases with impaired renal function, and patients mostly present with hallmarks of kidney injury, such as albuminuria and abnormal urinary sediment [1]. In recent years, the incidence of CKD has increased along with the rising incidence of basic diseases, such as diabetes mellitus and hypertension; especially the number of patients with end-stage renal disease has significantly increased [2], which seriously endangers the health of Chinese residents. Early detection and early diagnosis are important measures to reduce the medical burden of CKD patients, while CT is the routine diagnostic modality for CKD, which has significant advantages of high resolution and can obtain information on tissue microcirculation of patients, providing a scientific basis for physicians to diagnose CKD [3]. However, subtle renal vessels are difficult to discern by CT, and perfusion scans need to be repeated many times with higher radiation doses, predisposing patients to adverse effects [4]. Compared with conventional CT, 640-slice CT can avoid the radiation dose from repeated scanning without moving the bed and at the same time acquire multi-directional and multi-angular precise images, clearly show the relationship between blood vessels and surrounding viscera, and improve the quality of the examination [5, 6]. At present, the diagnostic value for CKD of 640-slice CT kidney scan and conventional CT scan had not been explored in the academia, so 120 CKD patients were selected for the study as the subjects to investigate the diagnostic efficacy of 640-slice CT kidney scan and conventional CT scan, with the results reported as follows.

## 2. Materials and Methods

### 2.1. Study Design

This retrospective study was conducted in our hospital from June 2019 to September 2019 to explore the diagnostic value of 640-slice CT kidney scan and conventional CT scan for CKD. It was a double-blind study, meaning that neither the subjects nor researchers understood the trial grouping, and the study designer was responsible for arranging and controlling the full trial.

### 2.2. General Data

A total of 120 CKD patients who received kidney plain scan plus enhanced examination in the CT room of the Medical Imaging Department of our hospital from June 2019 to September 2019 were selected and randomly divided into the experimental group (*n* = 60) and the control group (*n* = 60). In the experimental group, there were 38 males and 22 females, the patients' mean age was (40.28 ± 5.19) years, mean body mass was (64.98 ± 2.65) kg, and BMI was (22.65 ± 2.14) kg/m^2^, and in the control group, there were 35 males and 25 females, the patients' mean age was (40.65 ± 5.13) years, mean body mass was (65.05 ± 2.74) kg, and BMI was (22.74 ± 2.23) kg/m^2^. No significant differences in the baseline data between the two groups were observed (*P* > 0.05), so these patients could be selected as the subjects.

All patients met the diagnosis criteria for CKD [7], had no mental illnesses, and could tolerate CT examination [8]. Taking the CKD glomerular filtration rate (GFR) calculated by the plasma clearance rate of 99mTc-DTPA nuclear medicine as the standard [9] and according to the practice guideline for chronic kidney disease and dialysis [10], the patients were divided into mild, moderate, and severe renal impairment. In the experimental group, 18 cases had mild renal impairment, 28 cases had moderate renal impairment, and 14 cases had severe renal impairment, and in the control group, 20 cases had mild renal impairment, 27 cases had moderate renal impairment, and 13 cases had severe renal impairment. For CKD stage 1, GFR = 30–45.5 ml/(min × 1.73 m^2^), meaning mild impairment; for CKD stages 2 and 3, GFR = 15–29.9 ml/(min × 1.73 m^2^), meaning moderate and severe impairment. Patients at stages 4 and 5 of CKD had a serious renal impairment and were not suitable for using the contrast agent, and thus they were excluded from the study. In addition, those who suffered from hearing disorder, language barrier, unconsciousness, mental illness, and other factors, who quit the treatment in the middle of the study, who had other severe organic diseases [11], who were pregnant or lactating women, and who were allergic to the contrast agent and infants were not included in the study.

### 2.3. Moral Consideration

The study met the principles of the World Medical Association Declaration of Helsinki (2013) [12] and was approved by the Hospital Ethics Committee. The patients understood the study objective, meaning, content, and confidentiality and signed the informed consent.

### 2.4. Methods

#### 2.4.1. Control Group

The patients were told to empty the stomach and hold the urine. They were in the supine position and kept smooth breathing, foot first was selected, and the parameters of Toshiba 64-slice CT scanner (NMPA (I) 20063300657) were set as follows: tube voltage of 120 kV, tube current of 310 mA, noise index of 8.63, speed of 0.6 s/circle, slice thickness of 5 mm, pitch of 0.984, and FOV of 36 cm × 36 cm. Low-concentration iso-osmotic non-ionic contrast medium, iodixanol (manufacturer: Jiangsu Hengrui Medicine Co. Ltd.; NMPA approval no. H20103675), was administered via intravenous injection through the right median cubital vein by a single-tube pressure syringe, with a total dose of 65 ml and a rate of 3.5 ml/s. After injection, enhanced scans in the cortical phase, myeloid phase, and secretory phase were performed, and the CT values were measured by the workstation.

#### 2.4.2. Experimental Group

Patients received CT plain scan first; after the range of 640-slice CT dynamic volume scan was determined, Toshiba 320/640 volume CT (NMPA (I) 20143303426) was used to determine the scan position of both kidneys according to the scout view, the detector effective width was ensured to an extent of containing bilateral whole kidneys, and the dynamic volume enhanced perfusion scan was performed with the following parameters: tube voltage of 100 kV, tube current of 50 mAs, rotation time of 0.5 s, collimation of 0.5 mm × 230, and slice thickness of 0.5 mm. Low-concentration iso-osmotic non-ionic contrast medium, iodixanol, was administered via intravenous injection through the right median cubital vein by a double-tube pressure syringe, with a total dose of 65 ml and a rate of 3.5 ml/s. After injection, enhanced scans in the cortical phase, myeloid phase, and secretory phase were performed, and the CT values were measured by the workstation.

### 2.5. Observation Criteria

After finishing the experiment, the experimental data and test data were collected to perform subjective scoring of the images, the effective radiation dose (dose-length product × *K* value, the dose-length product was generated automatically by the computer, and the K value referred to the *European Guidelines on Quality Criteria for Computed Tomography* [13]), signal-to-noise ratio (SNR), and contrast-to-noise ratio (CNR) were calculated, and the imaging quality and effective radiation dose were compared between the two modalities. The CT values were calculated by the workstation, and the relationship between the CT values from 640-slice CT scan and conventional CT scan and kidney injury was analyzed. The subjective scoring criteria for image quality are shown in Table 1.

### 2.6. Statistical Processing

In this study, the data processing software was SPSS18.0, and the picture drawing software was GraphPad Prism 7 (GraphPad Software, San Diego, USA). The data included enumeration data and measurement data, tested by *X*^2^ test and *t*-test. The differences were considered statistically significant at *P* < 0.05.

## 3. Results

### 3.1. Between-Group Comparison of Imaging Quality

Compared with the control group, the image quality of 640-slice CT scan conducted in the experimental group was significantly better (*P* < 0.05) (see Table 2 and Figure 1).

The SNR was significantly higher in the experimental group than in the control group (15.98 ± 0.65 vs 12.12 ± 0.47, *P* < 0.001).

The CNR was significantly higher in the experimental group than in the control group (30.98 ± 2.68 vs 12.98 ± 1.58, *P* < 0.001).

### 3.2. Between-Group Comparison of Effective Radiation Doses

The effective radiation doses of the experimental group and the control group were, respectively, (1.89 ± 0.32) mSv and (3.26 ± 0.47) mSv, indicating that the dose was significantly lower in the experimental group than in the control group (*t* = 18.664, *P* < 0.001).

### 3.3. Analysis of Relationship between CT Values of the Two Groups and Kidney Injury

The correlation analysis showed that the relationship between the sum of CT values in the cortical phase of both kidneys and kidney injury in the experimental group was *r* = 0.835, *P* < 0.001.  Figure 2 shows the CT values of the two groups.

In the experimental group, the CT values of patients with mild, moderate, and severe renal impairment in the cortical phase were, respectively, (133.43 ± 9.80) HU, (125.65 ± 9.55) HU, and (87.66 ± 9.65) HU, and in the control group, the CT values of patients with mild, moderate, and severe renal impairment in the cortical phase were, respectively, (145.98 ± 9.55) HU, (140.65 ± 9.57) HU, and (102.98 ± 9.57) HU.

In the experimental group, the sums of CT values of patients with mild, moderate, and severe renal impairment in the cortical phase were, respectively, (288.98 ± 9.65) HU, (245.98 ± 9.65) HU, and (170.98 ± 9.50) HU, and in the control group, the sums of CT values of patients with mild, moderate, and severe renal impairment in the cortical phase were, respectively, (310.98 ± 9.54) HU, (279.65 ± 9.10) HU, and (200.98 ± 9.55) HU.

## 4. Discussion

There are many kinds of kidney diseases, and the common ones include calculus, inflammation, tuberculosis, tumors, and congenital dysplasia [14, 15]. The incidence of chronic kidney disease (CKD) in China is about 10.8%. Previously, GFR was an important criterion for the diagnosis of CKD, but the kidney is an important organ to maintain a stable environment in the human body with extremely strong metabolic function and compensatory function, so for some patients in the early stage of mild renal impairment, early CKD cannot be effectively diagnosed because the change in blood creatinine concentration is slight and the GFR calculated from creatinine is also not significantly abnormal. Given that physiopathological changes in the kidney are closely related to blood flow, CT has become the most effective modality for diagnosing CKD [16]. In recent years, studies have shown that the plasma clearance of non-ionic contrast agents is close to inulin, so the metabolism of non-ionic contrast agents in the kidney can be observed with CT [17]. However, CT perfusion scan requires multiple repeated scans with a higher radiation dose and is not suitable for patients with serious renal injury [18], so the application of CT enhanced scan in the diagnosis of CKD is limited. Compared with conventional CT, 640-slice CT is more suitable for older patients, severe patients, and those with poor compliance [19, 20], which uses a 16 cm wide detector with a fast scanning speed, can obtain 0.5 mm slice thick isotropic images and zero phase delay information of organ, and has more diversified post-processing methods, and after the scan, the scanning level can also be corrected by software to improve the precision of the measurements. Therefore, 640-slice CT has a broader scope of application and can meet the shift in imaging diagnosis of CKD from morphological diagnosis to functional diagnosis. The study results showed that SNR and CNR of 640-slice CT scan in the experimental group were significantly better than those of conventional CT in the control group (*P* < 0.05). Noise and CNR are the important criteria for evaluating the image quality, with higher CNR indicating better image quality. Also, the experimental group obtained a higher subjective score, proving that the image quality of 640-slice CT is more stable. In addition, the effective radiation doses obtained by the experimental group and the control group were, respectively, (1.89 ± 0.32) mSv and (3.26 ± 0.47) mSv, demonstrating that 640-slice CT can reduce the scanning radiation dose while obtaining images with better quality, which is conducive to reducing the adverse risks of ionizing radiation to the patients and presents exact application value.

Scholars You et al. showed that the blood flow of renal cortex obtained by 640-slice CT after scanning with reduced radiation dose was not significantly different from that of the conventional dose group, indicating that further reducing radiation dose still did not affect the accuracy of 640-slice CT, so this examination modality can effectively reflect the situation of the renal cortex [21]. Renal cortical blood flow accounts for 90.00% of the total renal blood volume, 94.00% of the glomeruli are located in the renal cortex, and the functional and morphological changes can reflect the degree of damage to the kidney, so under the circumstances of consistent image acquisition time and location in the cortical phase, changes in the degree of cortical enhancement (CT values) can reflect differences in the filtration function of the kidney [22, 23], thereby providing a basis for the diagnosis of CKD. Compared with conventional CT, 640-slice CT has the same renal phase at the time of measurement, so the acquired CT values in the cortical phase are more precise [24]. In this study, the CT value in the cortical phase and the sum of CT values in the cortical phase were lower in the experimental group than in the control group, and the correlation analysis showed that the relationship between the sum of CT values in the cortical phase of both kidneys and kidney injury in the experimental group was *r* = 0.835, *P* < 0.001, proving significant correlation of the sum of CT values in the cortical phase of both kidneys and kidney injury in the experimental group. Scholars Hori et al. reported that Pearson analysis of CT contrast-enhanced scan correlation measures can similarly yield a correlation between the sum of CT values in the cortical phase of both kidneys and renal injury [25], but with the overall consideration of conditions such as image quality and scanning radiation dose, 640-slice CT still presents significant advantages, making this diagnostic modality the most sensitive method of renal vascular examination at the current stage, which is beneficial for enhancing the efficiency of clinical diagnosis of CKD and improving the precision of diagnosis.

In conclusion, both 640-slice CT kidney scan and conventional CT scan can be used in the diagnosis of CKD. The 640-slice CT has a lower radiation dose, better image quality, and higher application value. Therefore, the study of 640-slice CT kidney scan can be deepened to provide more references for the clinic and increase the application frequency of 640-slice CT kidney scan.

## Figures and Tables

**Figure 1:** Between-group comparison of (a) SNR and (b) CNR ($\bar{x}\pm s$).

**Figure 2:** Analysis of relationship between CT values of the two groups and kidney injury ($\bar{x}\pm s$, HU). (a) The CT values in the cortical phase. (b) The sum of CT values in the cortical phase.

**Table 1:** Subjective scoring criteria for image quality.

Grade	Scoring criteria
1	With clear anatomical details and structures, sharp image edges, and no artifacts or obvious noise, the images could be used for diagnosis directly

2	With fairly clear anatomical details and slight artifacts and noise, the anatomical structures of the images could meet the diagnostic requirements

3	Fairly clear anatomical structures, vague image edges, and fairly obvious artifacts and noise

4	Unrecognizable fine anatomical structures, unclear images, and extremely obvious artifacts and noise

**Table 2:** Between-group comparison of subjective scores ($\bar{x}\pm s$, points).

Group	Plain scan	Cortical phase	Myeloid phase	Secretory phase
Experimental	1.38 ± 0.49	1.85 ± 0.65	2.10 ± 0.83	2.13 ± 0.59
Control	1.32 ± 0.47	2.37 ± 0.75	2.43 ± 0.69	2.65 ± 0.79
*t*	0.685	4.058	2.368	4.085
*P*	0.495	<0.001	0.020	<0.001

## Data Availability

The data used to support the findings of this study are available on reasonable request from the corresponding author.
